# Deep Learning for Ocular Disease Recognition: An Inner-Class Balance

This article has been retracted.

**DOI:** 10.1155/2022/5007111

**Published:** 2022-04-28

**Authors:** Md Shakib Khan, Nafisa Tafshir, Kazi Nabiul Alam, Abdur Rab Dhruba, Mohammad Monirujjaman Khan, Amani Abdulrahman Albraikan, Faris A. Almalki

**Affiliations:** ^1^Department of Electrical and Computer Engineering, North South University, Bashundhara, Dhaka 1229, Bangladesh; ^2^Department of Computer Science, College of Computer and Information Sciences, Princess Nourah Bint Abdulrahman University, P.O. Box 84428, Riyadh 11671, Saudi Arabia; ^3^Department of Computer Engineering, College of Computers and Information Technology, Taif University, P.O. Box 11099, Taif 21944, Saudi Arabia

## Abstract

It can be challenging for doctors to identify eye disorders early enough using fundus pictures. Diagnosing ocular illnesses by hand is time-consuming, error-prone, and complicated. Therefore, an automated ocular disease detection system with computer-aided tools is necessary to detect various eye disorders using fundus pictures. Such a system is now possible as a consequence of deep learning algorithms that have improved image classification capabilities. A deep-learning-based approach to targeted ocular detection is presented in this study. For this study, we used state-of-the-art image classification algorithms, such as VGG-19, to classify the ODIR dataset, which contains 5000 images of eight different classes of the fundus. These classes represent different ocular diseases. However, the dataset within these classes is highly unbalanced. To resolve this issue, the work suggested converting this multiclass classification problem into a binary classification problem and taking the same number of images for both classifications. Then, the binary classifications were trained with VGG-19. The accuracy of the VGG-19 model was 98.13% for the normal (N) versus pathological myopia (M) class; the model reached an accuracy of 94.03% for normal (N) versus cataract (C), and the model provided an accuracy of 90.94% for normal (N) versus glaucoma (G). All of the other models also improve the accuracy when the data is balanced.

## 1. Introduction

The diagnosis of ocular pathology using fundus images is a significant difficulty in health care [1]. Ocular disease refers to any condition or disorder that interferes with the eye's capacity to operate correctly or has a detrimental impact on the eye's visual acuity [2]. Almost everyone suffers from vision problems during their lifetime. Some are minors that do not appear on claims or are easily treated at home, while others need a specialist's attention [3]. Globally, fundus disorders are the primary cause of blindness in humans. Diabetic retinopathy (DR), glaucoma, cataract, and age-related macular degeneration are the most common ocular illnesses (AMD). According to linked studies, more than 400 million individuals will have DR by 2030 [4]. These ocular illnesses are becoming a major global health concern. Most significantly, the ophthalmic illness is incurable, and it might result in permanent blindness. Early identification of these disorders helps avoid vision impairment in clinical circumstances. Nevertheless, there is a major disparity between the number of ophthalmologists and the number of patients. Furthermore, manually examining the fundus is time-consuming and vastly dependent on ophthalmologists' experience. This complicates large-scale fundus screening. As a result, automated computer-aided diagnostic techniques for detecting eye disorders are vital. This is a common misunderstanding [4].

The frequency of eye diseases varies widely around the world, depending on factors such as age, gender, occupation, lifestyle, economic level, hygiene, customs, and conventions. A study of tropical populations compared with temperate regions shows that tropical populations have increased prevalence of irresistible eye infections due to natural components such as dust, humidity, daylight, and other factors [5]. Also, between emerging and developed countries, eye illnesses manifest differently within communities. Many underdeveloped countries, particularly in Asia, have high levels of ocular morbidity which are underdiagnosed and untreated [6]. The number of people with vision impairments is projected to be 285 million worldwide, of whom 39 million are blind and 246 million have impaired vision [7]. According to the World Health Organization (WHO), around 2.2 billion people suffer from some form of close-up or distance vision problem [8]. Half of these scenarios, according to estimates, might have been prevented or healed. There are 1 billion people who have moderate-to-severe distance vision impairment or blindness as a result of uncorrected refractive errors (88.4 million), cataract (94 million), glaucoma (7.7 million), corneal opacities (4.2 million), diabetic retinopathy (3.9 million), and trachoma (2 million), as well as those who have near vision impairment as a result of uncorrected presbyopia (826 million) [9]. Globally, uncorrected refractive errors, cataracts, age-related macular degeneration, glaucoma, diabetic retinopathy, corneal opacity, trachoma, hypertension, and so forth are the major causes of visual impairment [10]. In Bangladesh, there has been very little research on the prevalence of blindness and visual impairment. The country is mainly populated by rural dwellers. Currently, over 80% of individuals living in metropolitan areas require medical care, with a fair lack of ophthalmology services. Despite the increasing number of establishments offering blindness services, the prevalence remains low [11]. According to the Bangladesh National Blindness and Low Vision Survey, 21.6% of Bangladesh's population has low vision, which is defined as having a visual acuity of fewer than 6 inches in one of the eyes. It is possible that the rising incidence of noncommunicable illnesses such as diabetes and smoking is contributing to Bangladesh's higher risk of visual loss [12]. The 2013 Urban Health Survey found that many of the poor individuals residing in slums have poor mental and physical health status [13]. This makes it important to provide comprehensive eye care services to these individuals at low or no cost. Deep-learning-based algorithms are becoming more prevalent in medical image analysis. Deep-learning-based models have been shown to perform well in different tasks like object detection, sentiment analysis [14], medical image classification [15], and disease detection [16]. The automatic identification of illnesses is a key step in reducing an ophthalmologist's workload. Deep learning and computer vision technologies can detect diseases without requiring manual intervention. Although many of these studies have shown promising results, only a few of them have been able to provide a complete diagnosis [17] of more than one eye sickness. Further research is needed to analyze the various aspects of fundus imaging [18] to properly diagnose different eye ailments. This paper proposes a system that can identify various types of eye diseases through deep learning. Another approach has been made with multilabel classification [19]. The datasets [20–22] of this ocular disease are highly imbalanced. Due to this imbalance, the accuracy of detection or classification of disease or even a normal image is relatively low. With such low accuracy, it is not ideal to use this approach in generalized classification tasks.

The aim of this work was to classify ocular diseases. The dataset used in this study was highly imbalanced and, with such a dataset, classifying any disease is not advisable. Because of this imbalance, a lot of fluctuation occurs during training, which is not ideal. This approach has been taken to tackle this problem by balancing the image between the two classes. Rather than using all the images and classifying all the diseases at once, we take two classes at a time and balance them by taking the same number of images from both classes and feeding them into a pretrained VGG-19 model.

As a result, this research first balanced the dataset by using the same amount of data for each class and training them using the pretrained VGG-19 architecture. First, we loaded the dataset and the corresponding image into the dataset by taking the same number of images for both classes. This work utilized the transfer learning method for the VGG-19 model. After we balanced the dataset properly, the accuracy of the individual class improved.

The remainder of the paper is organized as follows: Section 2 shows the relevant work for this study. In Section 3, all the tools and methods are discussed thoroughly.  Section 4 discusses the outcomes and performance analysis of our work, and then our work concludes in Section 5.

## 2. Related Work

Different approaches have been initiated in relation to the classification of ocular diseases. The authors in [23] suggested a two-stage technique for performing optical disc (OD) localization using convolutional neural networks (CNN) on fundus pictures. Another research found that researchers introduced automatic ocular illness categorization models [24] that are based on knowledge distillation. This system is constructed by sequentially training and optimizing two deep networks. Lee et al. [25] proposed ReLayNet, a fully convolutional deep network for segmenting retinal layers and fluids from OCT scans. This technique uses an encoder-decoder network to segment semantic information from OCT scans. Researchers [26] developed a way to diagnose distinct retinal diseases by using optical coherence tomography. The pixel-wise classification of OCT scans was performed [27] using convolutional neural networks with dilated convolution filters. Based on 400 OCT scans of patients with varying stages of age-related macular degeneration, the model's performance was evaluated. On OCT images, Hu et al. [28] suggested a CNN-based approach for detecting intraretinal fluid. Using 1,289 OCT scans, the CNN model was trained, and the segmented pictures received a Dice score of 0.911 upon cross-validation. The authors [29] introduced a supervised learning technique to a unique convolutional multitask architecture. This model has been trained to execute three tasks at the same time: brilliant lesion segmentation, red lesion segmentation, and lesion detection. It performed well, with an AUC of 0.839. A retinal vascular segmentation algorithm [30] is proposed based on fully connected conditional random fields and a convolutional neural network (CRFs). The model's accuracy and effectiveness were tested using color fundus pictures from the STARE [31] and DRIVE [32] datasets. Khan et al. [33] developed a deep-learning-based method to automate the identification of diabetic macular edema and diabetic retinopathy. This challenge was completed with the help of a neural-network-based picture categorization model that was optimized. Researchers in [34] proposed the use of deep-learning-based approaches (GONs) to detect glaucomatous optic neuropathy. They also included pictures of the colors of the fundus. For training their classification model, researchers used over 8,000 images of the color fundus. A model with a sensitivity score of 95.6 percent and a specificity score of 92.2 percent yields an AUC value of 0.98. Using optical coherence tomography (OCT) pictures, this work [35] was able to diagnose distinct retinal diseases. Convolutional neural networks, such as GoogLeNet, were tuned to produce this approach. In the dataset used in this study, there were four classifications, including dry age-related macular degeneration, diabetic macular edema, and no pathology. Also, the authors in [36] used VGG-19 to detect cataracts by using color fundus images. Researchers in [37] investigated the principles of experimentation involved in evaluating the various methods. The authors in [38] implemented the study of various deep learning models for eye disease detection where several optimizations were performed. In [39], the authors did some benchmark experiments on it using some state-of-the-art deep neural networks. In [3–41], the authors used various models and algorithms for machine learning and deep learning.

## 3. Methodology

### 3.1. Proposed System

The dataset was balanced by using the same amount of data for each class in this paper, and the classes were trained using the pretrained VGG-19 architecture. We began by loading the dataset and corresponding images into the model, using the same number of images for both classes. The transfer learning method was used in this work for the VGG-19 model. The accuracy of the individual classes improved after we properly balanced the dataset. The work attempted to identify the correct class after training. The suggested system's workflow is represented in Figure 1.

Figure 1 illustrates the steps involved in the research. It shows that all those left and right eyes images have been trained individually by applying the pretrained VGG-19 model. Following training, they were classified as either Class 1 (disease) or Class 2 (normal).

### 3.2. Dataset

ODIR (Ocular Disease Intelligent Recognition) is the dataset [42] used in this study. This dataset is one of the most comprehensive resources available to the public on Kaggle for detecting eye diseases. The fundus images in this dataset are divided into eight categories of ocular disease classification. These categories include seven disease classes, that is, normal (N), myopia (M), hypertension (H), diabetes (D), cataract (C), glaucoma (G), age-related macular degeneration (A), and other abnormalities/diseases (O). This dataset contains 5000 color fundus photographs, which are divided into training and testing subsets. A little more than 3500 cases are used for training and the rest for testing. For this work, all images were resized to 224 × 224. Detailed information regarding image distributions for the ODIR dataset can be found in Table 1, and some sample images of the dataset can be viewed in Figure 2. Detailed information regarding this distribution of images is given in Figure 3.

The bar chart of the dataset is shown in Figure 2. The number of patients is shown on the *x*-axis, and the disease categories are shown on the *y*-axis. The bar chart represents the training cases of each class which were given in the dataset. According to the chart, it is shown that the normal (N) class has the highest number of patient cases, which is 1135, and the second highest case is from the diabetes (D) class. After that, it is shown that the hypertension (H) classes have the lowest patient cases.

A glimpse of the dataset is given in Figure 3. These are the fundus images from the dataset. A left label indicates the left eye, and a right label indicates the right eye.

### 3.3. Convolutional Neural Network

The convolutional neural network shows exceptional performance in image classification [43] and object recognition [44] applications. CNNs (convolutional neural networks) are one of the machine-learning methods for developing Multilayer Perceptrons (MLPs) designed to process two-dimensional data. CNNs are deep neural networks because they have multiple ways of combining image data in a network, which makes them a type of deep neural network. In CNNs, convolution is used as the basis for the algorithm. The CNN algorithm has multiple layers: convolution operations, activation layers, pooling layers, and flattening layers.

(1) $$\begin{array}{c} \text{Convolution Operation},C\left(i,j\right)=\;\left(I*K\right)\left(i,j\right)=\sum m\sum n\times I\;\left(m,n\right)K\left(i-m,j-n\right),\\ \text{Activation Layer},\mathrm{Sigmoid}\;S\left(x\right)=\frac{1}{1\;+\;e^{-x}}. \end{array}$$

### 3.4. Transfer Model

The transfer learning [19] technique refers to the use of a model created for one task as the basis for a model for another task. Deep learning models can be developed and implemented more effectively using transfer learning. Due to deep learning's increasing importance in tackling a wide variety of issues in fields such as computer vision (CV), we should expect to see more components of transfer learning. Transfer learning is only effective when the first model's characteristics learned on its first task are generalized and transferable to the second task. In this work, we used the pretrained VGG-19 model.

### 3.5. VGG-19

Deep neural networks have aided in a number of breakthroughs in image classification. Many other visual recognition tasks have benefited from these advanced models as well. Therefore, as time passes, we tend to deepen and solve more challenging tasks and improve our accuracy. As we progress deeper into neural networks, however, training gets harder and accuracy degrades as well. By implementing VGG-19 [20], these issues are being addressed. VGG-19 is a CNN-based model that uses 3 × 3 filters with a single stride and always employs the same padding and maxpooling layers of 2 × 2 filters with a stride of 2, instead of having a huge number of hyperparameters. In the architecture, the convolution and maxpooling layers are organized in a similar manner. There are two FC layers in the model. There are more than 138 million trainable parameters in this VGG-19 network, which is a large network.  Figure 4 depicts the VGG-19 network architecture.

After the classification layer, which included a densely connected classifier and a dropout layer, a series of convolutional layers were applied (conv1, conv2, conv3, conv4, and conv5). Each neuron in a dense layer is connected to all the neurons in the preceding layer. Compared with a convolutional layer, a densely connected layer learns from the previous layer's features. How the densely connected layer is activated must be specified.

### 3.6. Implementation Details

The model is configured to use the Adam optimizer and a binary cross-entropy loss function. Additionally, the sigmoid activation function is used. All experiments were carried out on Google Colab. After we hadd selected those parameters, we ran the model through 20 iterations on the training data. Finally, we evaluated the model on the test set.

## 4. Results and Analysis

### 4.1. Overview of Outcomes

Based on our research, we solved the class imbalance problem by taking the same number of images. There was a huge disparity between the classes in the ODIR dataset. By following this method, we are able to significantly improve our accuracy when the number of images is much lower. The relative metrics, accuracy loss graphs, and other equivalent indications of the performance evaluation methodologies were then examined and graphically shown. Using the VGG-19 architecture, we demonstrated our model's ability to accurately predict a particular condition. We used the confusion matrix on the test to show how accurate this model can predict.

### 4.2. Performance Evaluation

In our experiment, the CNN-based architecture VGG-19 was used to assess model performance. In the data sequencing and splitting part, first the image is taken from the dataset and the data are converted into train labels and target labels. The scikit-learn library's training-test split method was used. The data were divided into a 70 : 30 ratio, with 70% of the data being utilized for training and 30% for testing. The performance metrics of both models are presented in this section, as well as their prediction capabilities. Here are some results for each class.

#### 4.2.1. Glaucoma (G) versus Normal (N)

In the dataset, we only have 207 cases of glaucoma. To balance this, we took 206 normal cases so that the model does not overfit. After sampling the data from the dataset, we passed the data into the pretrained VGG-19 and got a training accuracy and loss.

In Figure 5, the initial accuracy for training was about 0.6 and the validation was 0.80. With each epoch, the accuracy of training and validation increases, and model loss decreases. After running 5 epochs, the model achieved training and validation accuracy of 0.97 and 0.90, respectively. Finally, the model training accuracy was about 1.0 and the validation accuracy was 0.92.

#### 4.2.2. Hypertension (H) versus Normal (N)

We only have 94 hypertension cases in the dataset; to balance this, we took 95 normal cases so that the model does not overfit. We sampled data from the dataset and fed them into a pretrained VGG-19 to calculate training accuracy and loss.

In Figure 6, the initial accuracy for training was about 0.59 and the validation was 0.64. With each epoch, the accuracy of training and validation increases, and model training and validation loss decreases. After running 5 epochs, the model achieved training and validation accuracy of 0.98 and 0.88, respectively. Finally, the model training accuracy was about 1.0 and the validation accuracy was 0.90.

#### 4.2.3. Pathological Myopia (M) versus Normal (N)

We only have 177 pathological myopia cases in the dataset, so we added 175 normal cases to ensure that the model does not overfit. To calculate training accuracy and loss, we sampled data from the dataset and fed them into a pretrained VGG-19.

In Figure 7, the initial accuracy for training was about 0.85 and the validation was 0.90. With each epoch, the accuracy of training and validation increases, and model loss decreases. After running 5 epochs, the model achieved training and validation accuracy of 0.96 and 0.98, respectively. Finally, the training accuracy was about 1.0 and the validation accuracy was 0.99.

#### 4.2.4. Other Diseases/Abnormalities (O) versus Normal (N)

We only have 177 pathological myopia cases in the dataset, so we added 175 normal cases to ensure that the model does not overfit. To calculate training accuracy and loss, we sampled data from the dataset and fed them into a pretrained VGG-19.

In Figure 8, the initial accuracy for training was about 0.4 and the validation was 0.65. With each epoch, the accuracy of training and validation increases, and model loss decreases. After running 5 epochs, the model achieved training and validation accuracy of 0.96 and 0.86, respectively. Finally, the training accuracy was about 1.0 and the validation accuracy was 0.90.

### 4.3. Evaluate Accuracy Metrics

For measuring goodness, we will use some metrics relating to accuracy in determining whether a particular image represents a disease. After all, we have used classification models. So we will use the most widely used metrics for classification problems.

#### 4.3.1. Training and Test Accuracy

While training our models using the training data, we will find out how much our model is learning from that training dataset. The main purpose of training accuracy is to extract the hyperparameters and to check whether our models have overfitting or underfitting issues.

(2) $$\begin{array}{c} \text{Accuracy}=\frac{\text{True Positive}\left(\text{ TP}\right)+\text{True Negative}\left(\text{TN }\right)}{\text{True Positive}\left(\text{TP}\right)+\text{True Negative}\left(\text{TN}\right)+\text{False Positive}\left(\text{ FP}\right)+\text{False Negative}\left(\text{ FN}\right)}. \end{array}$$

When we are done with training our models using our training dataset and we have also cross-checked that our models are doing well in the validation dataset, only then can we go for the test accuracy, which is the final accuracy of our models. When mentioning accuracy in our report, we mean test accuracy.

#### 4.3.2. Precision

Sometimes accuracy alone is not enough. We just cannot say that our model is very accurate by only looking at the accuracy, because, in this project, we have to classify both diseases and nondiseases correctly. In terms of deep learning, we can say that those who have a disease are called “positive” and those who do not have a disease are called “negative.” Precision gives a clear view of how many of the positive-meaning disease patients are identified correctly among the entire dataset.

(3) $$\begin{array}{c} \text{Precision}=\frac{\text{True Positive}\left(\text{TP}\right)}{\text{True Positive}\left(\text{TP}\right)+\text{False Positive}\left(\text{FP}\right)}. \end{array}$$

#### 4.3.3. Recall

Sometimes even precision is not enough. For example, if the dataset is highly biased towards one target, recall provides the number of correctly classified true positives, meaning those people who are actually diseased and our model has predicted that they are diseased.

(4) $$\begin{array}{c} \text{Recall }=\frac{\text{True Positive}\left(\text{TP}\right)}{\text{True Positive}\left(\text{TP}\right)+\text{False Negative}\left(\text{FN}\right)}. \end{array}$$

This recall is the most important metric of our research project, because if we have a poor recall, then our model can predict a diseased person incorrectly.

#### 4.3.4. F1 Score

The F1 score is called the harmonic mean of precision and recall. So if someone claims to give equal priority to precision and recall, then he/she can focus on the F1 score. In this study, our second highest priority after the recall is the F1 score.

(5) $$\begin{array}{c} F1\text{ Score}=2\times \frac{\text{Precision }\times \text{Recall}}{\text{Precision}+\text{Recall}}\text{.} \end{array}$$

Once the model has been trained, we evaluate it on a test set.  Table 2 represents the accuracy of the model. According to the accuracy history of the test set, the N against C class has an accuracy of 0.940, and the N against H class has an accuracy of 0.889. Further, we achieved an accuracy of 0.861 for N versus O, 0.866 for N versus A, 0.981 for N versus M, and 0.909 for N versus G. Thus, comparing each class to the typical class, the following table reveals that N versus M earned the highest accuracy score.

The test set accuracy is not enough to determine whether an image has a disease or not. So, to make it more accurate, we evaluate the test set on the various performance metrics. For this work, the metrics used were precision, recall, and F1 score.  Table 3 shows the level of accuracy attained by these metrics.

In Table 3, VGG-19 is used to determine if an eye has a normal fundus (N) or another class of disease. Here, 0 represents a normal fundus and 1 represents a diseased fundus. After implementing it with the model, we can see that almost every result is satisfactory, but we found a bit higher precision and recall score after classifying the normal (N) class with the cataract (c) class. In Table 3, we note that N has a precision of 0.92, a recall of 0.93, and an F1 score of 0.92, while C has a precision of 0.96, a recall of 0.95, and an F1 score of 0.95. Furthermore, in the N versus M class, the precision for the normal class is 1.00, the recall is 0.96, and the F1 score is 0.98. On the other hand, the precision for pathological myopia (M) is 0.97, the recall is 1.00, and the F1 score is 0.98.

### 4.4. Confusion Matrix

The performance of classification models has been assessed by the confusion matrix for a given dataset. Only if the true values of the test data were known could it be determined. A matrix in which predicted and actual values are separated, as well as the total number of forecasts, has two dimensions. A true value is determined by the observational data, whereas a projected value is determined by the model.

For some confusion matrices of classification, Figure 9 shows the N versus H class. It is shown that the implemented model VGG-19 can accurately classify 54 true positive (TP) images and 75 true negative (TN) images. The model misclassified some images too; the model predicted 12 false positives (FPs) and 4 false negatives (FNs).

Figure 10 shows the N versus G class. It is shown that the implemented model VGG-19 can accurately classify 93 true positive (TP) images and 128 true negative (TN) images. However, the model misclassified some images too; the model predicted 18 false positive (FP) images and 4 false negative (FN) values.

Figure 11 shows the N versus M class. It is shown that the implemented model VGG-19 can accurately classify 119 true positive (TP) images and 144 true negative (TN) images. However, the model misclassified some images too; the model predicted five false positive (FP) images and zero false negative (FN) values.

Figure 12 shows the N versus C class. It is shown that the implemented model VGG-19 can accurately classify 77 true positive (TP) images and 128 true negative (TN) images. However, the model misclassified some images too; the model predicted six false positive (FP) images and seven false negative (FN) values.

### 4.5. Detection of Each Classification

After training the VGG-19 model, we checked if it could easily identify images as normal or diseased. The detection of images is shown in Figures 13 and 14. It is clear that our model performs very well and can accurately predict the disease image and the nondisease image.

In Figures 13 and 14, we took random images from the test set and tried to see how our model could predict normal or disease. All the pictures showed that VGG-19 correctly identified which dermoscopic image was diseased or normal. With such a huge number of parameters, our model can predict as accurately as we expected, and this is clearly understandable, so VGG-19 performed appropriately in detecting ocular images.

### 4.6. Model Comparison

The pretrained model used in this study was compared to some referenced publications. In Table 4, we compare some works which have used different types of models for ocular diseases recognition.

The main difference is that most of the work trains all the classes together, whereas we train all the classes individually. From the above table, it is shown that VGG architecture is used mostly in ocular disease recognition tasks where they get less than 90% accuracy. Using VGG-19, this work is supposed to have a higher accuracy than the others, which is 97.94%. In our work, we also used the same VGG-19 which came up with 98.10% accuracy, slightly higher than the previously mentioned work. Researchers also implemented EfficientNet and DenseNet architectures and achieved comparatively less accuracy, which is nearly 86–87%. Among all these works mentioned above, our outcome shows a more accurate and precise view in classifying ocular diseases.

## 5. Conclusion

In this study, the model VGG-19 was used to classify the various types of ocular diseases, which predicted whether an eye has any disease or a normal fundus. Also, the performance is much better than expected. This work achieved the highest accuracy for normal versus myopia, which is 98.10%, and also got a 94.03% accuracy for the normal versus cataract class. Furthermore, we got a 90.94% accuracy rate for the normal versus glaucoma class. The proposed strategy surpasses existing CNN-based ocular disease classification models while requiring less latency. It is also easily adaptable to different sorts of medical image-based illness categorization. Furthermore, the VGG-19 model may be utilized to create a consumer-genuine ocular illness categorization system. The most appealing thing about this method is that it can be easily applied to other types of medical image-based disease classification. Moreover, ocular image segmentation could be applied to this work. Research can use generative adversarial networks (GANs) to produce similar ocular disease images to solve the imbalance problem. Furthermore, a system like this will be extremely useful to medical experts and will change the area of eye illness diagnostics. However, we feel that it can still be a useful model and that there are opportunities to enhance it with more studies in the near future and more exploration.

## Figures and Tables

**Figure 1:** An illustration of the proposed method.

**Figure 2:** Distribution of the dataset represented as a bar chart.

**Figure 3:** A sample view of the ODIR dataset [42].

**Figure 4:** VGG-19 architecture [20].

**Figure 5:** Model accuracy and loss for N versus G.

**Figure 6:** Model accuracy and loss for N versus H.

**Figure 7:** Model accuracy and loss for N versus M.

**Figure 8:** Model accuracy and loss for N versus O.

**Figure 9:** Confusion matrix for N versus H classification.

**Figure 10:** Confusion matrix for N versus G classification.

**Figure 11:** Confusion matrix for N versus M classification.

**Figure 12:** Confusion matrix for N versus C classification.

**Figure 13:** Prediction of normal (N) and glaucoma (G) classes with VGG-19 model.

**Figure 14:** Prediction of normal (N) and cataract (C) classes with VGG-19 model.

**Table 1:** Distribution of images in the ODIR dataset.

No. of classes	Labels	Training cases
1	Normal (N)	1135
2	Diabetes (D)	1131
3	Glaucoma (G)	207
4	Cataract (C)	211
5	Age-related macular degeneration (A)	171
6	Hypertension (H)	94
7	Pathological myopia (M)	177
8	Other diseases/abnormalities (O)	944

**Table 2:** The outcome results of test accuracy.

Classification	Test accuracy
N versus C	0.940
N versus H	0.889
N versus O	0.861
N versus A	0.866
N versus M	0.981
N versus G	0.909
N versus D	0.868

**Table 3:** Performance metrics of each class.

	Class	Precision	Recall	F1 score
N versus C	0	0.92	0.93	0.92
	1	0.96	0.95	0.95
N versus H	0	0.93	0.82	0.87
	1	0.86	0.95	0.90
N versus O	0	0.97	0.74	0.84
	1	0.80	0.98	0.88
N versus A	0	0.90	0.81	0.85
	1	0.84	0.92	0.88
N versus M	0	1.00	0.96	0.98
	1	0.97	1.00	0.98
N versus G	0	0.96	0.84	0.89
	1	0.88	0.97	0.92
N versus D	0	0.91	0.84	0.87
	1	0.86	0.92	0.89

**Table 4:** Comparison among different approaches.

Paper reference	Model name	Accuracy (%)	Our work
Paper [1]	VGGNet	89.75	**(VGG-19)** 98.10%
Paper [36]	VGG-19	97.94	
Paper [37]	VGG-16	81.76	
Paper [38]	EfficientNetB5	87.25	
	EfficientNetB6	86.52	
	DenseNet169	86.76	
Paper [39]	VGG-16 (off-site)	85.4	
	VGG-16 (on-site)	86.28	

## Data Availability

The data used to support the findings of this study are freely available at https://www.kaggle.com/andrewmvd/ocular-disease-recognition-odir5k.
